# Amelioration of Experimentally Induced Arthritis by Reducing Reactive Oxygen Species Production through the Intra-Articular Injection of Water-Soluble Fullerenol

This article has been retracted.

**DOI:** 10.3390/nano9060909

**Published:** 2019-06-23

**Authors:** Wen-Shuo Kuo, Chia-Tse Weng, Jian-Hua Chen, Chao-Liang Wu, Ai-Li Shiau, Jeng-Long Hsieh, Edmund Cheung So, Po-Ting Wu, Shih-Yao Chen

**Affiliations:** 1 School of Chemistry and Materials Science, Nanjing University of Information Science and Technology, Nanjing 210044, China; wskuo88@gmail.com; 2 School of Environmental Science and Engineering, Nanjing University of Information Science and Technology, Nanjing 210044, China; 3 Center for Micro/Nano Science and Technology, National Cheng Kung University, Tainan 701, Taiwan; 4 Department of Internal Medicine, National Cheng Kung University Hospital, College of Medicine, National Cheng Kung University, Tainan 701, Taiwan; ctweng@mail.ncku.edu.tw; 5 Department of Anesthesia, An Nan Hospital, China Medical University, Tainan 709, Taiwan; aptx4869jfk@gmail.com; 6 Department of Anesthesia, China Medical University, Taichung 404, Taiwan; 7 Department of Biochemistry and Molecular Biology, College of Medicine, National Cheng Kung University, Tainan 701, Taiwan; wumolbio@mail.ncku.edu.tw; 8 Department of Microbiology and Immunology, College of Medicine, National Cheng Kung University, Tainan 701, Taiwan; alshiau@mail.ncku.edu.tw; 9 Department of Nursing, College of Nursing, Chung Hwa University of Medical Technology, Tainan 717, Taiwan; pipi58871053@yahoo.com.tw; 10 Graduate Institute of Medical Sciences, Chang Jung Christian, Tainan 711, Taiwan; 11 Department of Orthopedics, College of Medicine, National Cheng Kung University, Tainan 701, Taiwan; 12 Department of Orthopedics, National Cheng Kung University Hospital Dou-Liou Branch, College of Medicine, National Cheng Kung University, Yunlin 640, Taiwan; 13 Department of Orthopedics, National Cheng Kung University Hospital, College of Medicine, National Cheng Kung University, Tainan 701, Taiwan; 14 Department of Biomedical Engineering, National Cheng Kung University, Tainan 701, Taiwan; 15 Medical Device R & D Core Laboratory, National Cheng Kung University Hospital, Tainan 701, Taiwan

**Keywords:** experimental arthritis, intra-articular injection, reactive oxygen species, rheumatoid arthritis, water-soluble fullerenol

## Abstract

Accumulated evidence suggests a pathogenic role of reactive oxygen species (ROS) in perpetually rheumatoid joints. Therefore, the application of radical scavengers for reducing the accumulation of ROS is beneficial for patients with rheumatoid arthritis (RA). We synthesized water-soluble fullerenols that could inhibit the production of ROS and applied intra-articular (i.a.) injection in an experimental arthritis model to examine the anti-arthritic effect of the synthesized compound. RAW 264.7 cells were used to examine the activity of the synthesized fullerenol. Collagen-induced arthritis (CIA) was induced in Sprague–Dawley rats by injecting their joints with fullerenol. The therapeutic effects were evaluated using the articular index as well as radiological and histological scores. Dose-dependent suppression of nitric oxide (NO) production caused by the fullerenol was demonstrated in the RAW 264.7 cell culture, thus confirming the ability of fullerenol to reduce ROS production. In the fullerenol-injected joints, articular indexes, synovial expression of ROS, histological and radiological scores, pannus formation, and erosion of cartilage and bone were all reduced. Moreover, interleukin (IL)-1β and vascular endothelial growth factor (VEGF) levels were reduced, and fewer von Willebrand factor (vWF)-stained areas were identified in the fullerenol-treated joints than in control joints. The i.a. injection of fullerenol for reducing ROS production can ameliorate arthritis in joints by suppressing pro-inflammatory cytokine production and the angiogenesis process. Thus, the i.a. injection of fullerenol for reducing the production of ROS can be used as a pharmacological approach for RA patients.

## 1. Introduction

Reactive oxygen species (ROS) have important physiological roles in maintaining cell redox status. They are necessary for regulating intracellular signaling pathways and transcription factors, such as nuclear factor-κB and hypoxia-inducible factor-1α, that are closely related to proinflammatory cytokine production and the angiogenesis process that is involved in the pathogenesis of rheumatoid arthritis (RA) [1,2]. In the synovial membrane of rheumatoid joints, the activation of leukocytes causes considerable consumption of oxygen, thus resulting in an increase in ROS release [3]. The first clinical evidence of the deleterious effect of ROS resulted from a trial involving RA patients. According to the evidence, the intra-articular (i.a.) injection of an enzyme-neutralizing superoxide anion can alleviate the pain in inflamed joints [4]. Accumulated evidence suggests a pathogenic role of ROS in perpetually rheumatoid joints. Therefore, the application of radical scavengers for reducing the accumulation of ROS is beneficial for treating RA.

Carbon and fullerene nanospheres have attracted considerable attention because of their pharmacological properties and biomedical applications [5,6]. In particular, a fullerene core reacts with free radical species, has an anti-oxidative capacity that is several hundred times higher than that of other antioxidants, and serves as a radical sponge in disease states related to ROS overproduction [5,7]. Although fullerene cores are insoluble in aqueous solutions, polyhydroxylated derivatives of fullerene (fullerenol) are soluble in hydroxyl groups. Thus, fullerenols provide water solubility while maintaining the affinity of their original skeletons for cellular lipid membranes [8]. Fullerenol acts as an effective catalyst in chemical and biochemical processes with identified pharmacological properties and exhibits no known toxicity toward animal or human cells [8,9,10,11]. Interestingly, a water-soluble derivative of fullerene entrapped in polyvinylpyrrolidone suppresses a joint through utilizing its anti-oxidative capacity [12]. In this study, synthesized water-soluble fullerenol was confirmed to have the ability to reduce ROS production. Moreover, two experimental arthritis models were used to examine the anti-arthritic effect of the i.a. or intraperitoneal (i.p.) administration of the synthesized fullerenol using prophylactic and therapeutic protocols.

## 2. Materials and Methods

### 2.1. Preparation and Characterization of Water-Soluble Fullerenol, C_60_(OH)_36_

Raw fullerene was obtained commercially (Sigma-Aldrich, St. Louis, MO, USA), and the C_60_(OH)_12_ precursor was produced, as previously described [13]. First, 30% hydrogen peroxide solution was added to the starting material, and the mixture was vigorously stirred at 60 °C under air. After cooling, a mixture of solvents comprising 2-propanol, diethyl ether, and hexane was added into the solution, which was subsequently centrifuged and decanted. The remaining solid was washed twice with diethyl ether through the general ultrasonic centrifugation and decantation procedures. Finally, the end product of water-soluble C_60_(OH)_36_ was obtained by drying the residue under vacuum at room temperature. The weight of the end product was calibrated through thermal gravimetric analysis. The morphology of the end product was observed using a high-resolution transmission electron microscope (HR-TEM, JEOL 3010, Akishima, Tokyo, Japan) at a resolution of approximately 1.08 ± 0.03 nm. The dynamic light scattering (DLS, Malvern Nano-ZS90, Worcestershire, West Midlands, UK) was also used to determine the size of nanomaterials. The exposed functional groups of the as-prepared nanomaterials were first examined through Fourier transform infrared (FTIR) spectroscopy (RX1, PerkinElmer, Waltham, MA, USA). Ultraviolet–visible (UV–Vis) spectroscopy of the nanomaterials was conducted using a spectrometer (U-4100, Hitachi, Chiyoda-ku, Tokyo, Japan). The number of hydroxyl groups was confirmed to be 36 based on the results provided by X-ray photoelectron spectrometry (XPS) results using a PHI 5000 spectrometer (VersaProbe, Chanhassen, MN, USA). A graph of the water-soluble C_60_(OH)_36_ is displayed in Figure 1.

### 2.2. Determination of ROS Reduction Ability

The reaction of C_60_(OH)_36_ with superoxide radicals was evaluated by examining the ability of C_60_(OH)_36_ to inhibit ROS production through in vitro phagocytosis of these particles by using a mouse macrophage line, RAW 264.7. In brief, the cells were placed in a 96-well microplate with a density of 1 × 10^4^ per well and were incubated with PBS or various concentrations of fullerenol for 2 h at 37 °C in a 5% CO_2_ incubator. The culture supernatants were replaced with fresh media, and the plates were continuously cultured for another 48 h in the presence of 1 µg mL^−1^ lipopolysaccharides (LPS, Sigma-Aldrich, St. Louis, MO, USA). The NO that had accumulated in the culture supernatants was measured using a colorimetric assay kit (Abcam, Cambridge, UK).

### 2.3. Induction of Mouse and Rat Collagen-Induced Arthritis (CIA)

The Institutional Animal Care and Use Committee of National Cheng Kung University approved the following animal experiments. Eight-week-old male DBA/1J mice housed under a specific-pathogen-free (SPF) condition were immunized intra-dermally (i.d.) with 100 µg of bovine type II collagen (Elastin Products Company, Owensville, MO, USA) in 50 µL of 0.1 M acetic acid emulsified with 50 µL of Freund’s complete adjuvant (Chondrex, Redmond, WA, USA) at the base of the tail on day 0. On day 21, the specimens received an i.p. booster of collagen without adjuvant, thus resulting in a more than 90% incidence of the development of arthritis [14,15]. Eight-week-old Sprague–Dawley male rats housed under the SPF condition were immunized i.d. on day 0 through an injection of 0.5 mL of 1:1 mixture of 400 µg of bovine type II collagen (Elastin Products Company, Owensville, MO, USA) with 0.1 M acetic acid and Freund’s complete adjuvant (Chondrex, Redmond, WA, USA) into four sites on the back. Booster doses were administered on day 7 with through injection of 0.25 mL of the same emulsion into the posterior aspects of the hip joints as described previously [14,16].

### 2.4. In Vivo Delivery of Synthesized Fullerenol 

On day 22, mice with CIA were divided into groups and received an i.p. injection of 30 µg of water-soluble C_60_(OH)_36_ or a control phosphate-buffered saline (PBS) injection (10 mice per group), as described previously [14]. For the i.a. injection, the ankle joints of the CIA rats were held in plantar flexion at an angle in the range of 15° to 20°; subsequently, a 31-gauge needle was mounted on a plastic syringe and inserted anterolaterally into the joint line at a distance of 1 to 2 mm from the lateral malleolus as described previously [16]. On the same day when they received the booster immunization using the prophylactic protocol, the right ankle joints of the remaining rats received 10 µM of water-soluble C_60_(OH)_36_, whereas the left ankles received a PBS injection to serve as the controls (16 joints per group). Another group of rats received 30 µM of water-soluble C_60_(OH)_36_ in their right ankles or a control PBS injection into their left ankles (16 joints per group) on day 10 after the development of arthritis after the therapeutic protocol was used. Moreover, similarly to the administering of the water-soluble C_60_(OH)_36_, 10 and 30 µM of unmodified (raw) fullerene was injected into the joints of CIA rats using the prophylactic and therapeutic protocols, respectively, and a PBS injection similarly served as the control.

### 2.5. Evaluation of Arthritis through Clinical, Radiological, and Histological Assessments

The clinical signs of mouse CIA were evaluated using scores from 0 to 3 for each paw, for a maximum of 12 points, as described previously [14]. Briefly, each limb was graded from 0 to 3 (0 = normal, 1 = slight swelling and/or erythema, 2 = pronounced swelling, 3 = ankylosis), giving a maximum score of 12 per mouse. The clinical evaluation of rat CIA was performed by calculating the articular index from 0 to 4, as described previously [17]. Briefly, the articular index was scored from 0 to 4 (0 = no swelling or erythema, 1 = slight swelling and /or erythema, 2 = low to moderate edema, 3 = pronounced edema with limited joint usage, 4 = excess edema with joint rigidity). Upon sacrifice of the rats on day 21, their ankles were removed for radiological examination. Radiographic scoring was performed by using imaging plates, and the radiographs were analyzed by a digital imaging system (Soredex, Tuusula, Finland). Radiographs were scored on a scale of 0 to 3 based on the joint space between the tibia and calcaneus, the tibia and talus, the talus and calcaneus. Then the graphs were scored for the degree of bony destruction from a 0 to 4 scale, assigning a point for erosion in the tibia, calcaneus, talus, and any one of the metatarsals. The soft tissue swelling was also scored on a scale of 0 to 3 (0 = no swelling, 1 = mild swelling, 2 = moderate swelling, 3 = severe swelling). All scores were summed up with a total scale from 0 to 10 [18]. The ankles were removed en bloc, fixed in formalin, decalcified, embedded in paraffin, sectioned, and subjected to hematoxylin and eosin (H&E) staining. The presence of synovial hyperplasia, cartilage erosion, and inflammatory infiltrates with leukocytes was evaluated and scored semiquantitatively on a scale of 0 to 2 for each item (0 = absent and normal, 1 = mild and slight, 2 = severe and pronounced), where the maximum score an ankle joint could receive was 6 (Figure 2) [16].

### 2.6. Immunohistochemical Staining and Enzyme-Linked Immunosorbent Assay (ELISA) 

After de-paraffinization and re-hydration, 5 µm synovial sections were stained with anti-nitrotyrosine (Abcam, Cambridge, UK) or anti-vWF antibody (DAKO, Agilent, Santa Clara, CA, USA), followed by horseradish-peroxidase-labeled secondary antibody (Jackson ImmunoResearch, West Grove, PA, USA) and substrate chromogen 3-amino-9-ethylcarbazole (Zymed Laboratories, South San Francisco, CA, USA), and expression intensities were quantified using the HistoQuest analysis software (TissueGnostics, Tarzana, CA, USA) as described previously [15]. The removed joints were skinned and further homogenized in 1 mL of radioimmunoprecipitation assay (RIPA) lysis buffer containing a protease inhibitor cocktail (Pierce Manufacturing, Appleton, WI, USA). Then, the concentrations of interleukin (IL)-1β, tumor necrosis factor (TNF), and vascular endothelial growth factor (VEGF) were measured using rat ELISA kits (R&D Systems, Minneapolis, MN, USA) according to the manufacturer’s protocol, as described previously [17].

### 2.7. Statistical Analysis 

Data are expressed in the mean ± standard error format. Differences in the articular indices and arthritis scores were calculated through repeated-measures analysis of variance. Other data were assessed using Student’s *t*-test. A *p*-value less than 0.05 was considered significant in this study.

## 3. Results and Discussion

The illustrative graph presented in Figure 1 features the water-soluble C_60_(OH)_36_ (fullerenol) in a circular-like shape with monodispersion, which was synthesized on the basis of a previous study [13], and the mean lateral size of a fullerenol molecule was approximately 1.08 ± 0.03 nm determined through the low-magnification (Figure 3A) and highly magnified HR-TEM images (Figure 3B). The crystallinity, which was favorable; lattice distance; and corresponding *d*-spacing of the fullerenol {$1\bar{1}00$} lattice fringes were also determined. However, the nanomaterials could form aggregation by hydrogen bonds in a pH 7.0 aqueous solution with the average size of approximately 125.7 nm by the DLS analysis (Supporting Information, Figure S1). In the UV–Vis absorption spectrum of fullerenol, it had no light absorption peaks and may be characterized by consequently strengthening light absorption with the longer wavelengths (>600 nm), evidencing peaks approximately 210 nm corresponded to the π–π* transition of aromatic C=C bonds. The n–π* transitions of the C=O shoulder appeared at approximately 319 nm; this indicated the π electron transition in fullerenol containing oxygen, whereas prominent absorbance bands were observed near 210 nm with a broad peak in the range of 190–580 nm, confirmed the existence of C_60_ (Figure 3C). This result is typically observed of aqueous dispersions of fullerenol. Further characterizations were performed through FTIR spectroscopy, and XPS [18] to confirm the identity of the as-prepared nanomaterials. FTIR spectroscopy was used to analyze the exposed functional groups of the as-prepared nanomaterials. The characteristic bands of the nanomaterials, including C–ONa (approximately 1014 cm^−1^), C–OH (approximately 1064 cm^−1^), C=O (approximately 1412 cm^−1^), C=C (approximately 1653 cm^−1^), and O–H (approximately 3238 cm^−1^), and the band of CO_2_ interference, were revealed the aromatic C=C bonds, and exposed hydroxyl and carbonyl groups (Figure 3D). The surface chemistry of the fullerenol, which typically contains predominately carbon atoms, was examined through XPS. The deconvoluted C(1s) spectra of the fullerenol presented a nonoxygenated C–C or C=C bond (286.1 eV), C–OH bond (286.9 eV), and C–O^−^ bond (288.1 eV), and the O(1s)–C(1s) ratio was approximately 37.1% (Figure 3E). The number of hydroxyl groups (C–OH) was confirmed to be 36 based on the results provided from the atomic ratios and bonding compositions of the fullerenol summarized in the table of Figure 3. On the basis of the aforementioned characterizations, the results confirmed that the fullerenol had been successfully synthesized. Moreover, in the culture experiment with RAW 264.7 cells, dose-dependent suppression of NO production was observed after the addition of various concentrations of fullerenol (Figure 4). This result confirmed the ability of fullerenol to reduce ROS production.

First, we injected fullerenol into the ankle joints of the rats with CIA on day 7 immediately after the second immunization. As presented in Figure 5A, compared with the control joints, the articular indexes of the fullerenol-injected joints were significantly lower. Compared with the PBS-injected joints, the fullerenol-treated joints exhibited significantly less synovial expression of nitrotyrosine, a product of tyrosine nitration mediated by ROS (Figure 5B). The fullerenol-injected joints exhibited less synovial inflammation, pannus formation, and erosion of cartilage and bone as well as significantly lower histological scores (Figure 5C). Moreover, less joint destruction and bone erosion were found in the radiographs of the fullerenol-injected joints, which had significantly lower radiological scores (Figure 5D). Further measurements of the proinflammatory cytokines in the CIA joints revealed significantly lower IL-1 levels in the fullerenol-treated joints than in the control joints (Figure 6A). However, there was no difference between the tumor necrosis factor (TNF) levels of the two groups (data not shown). In the angiogenesis process, there were significantly lower VEGF levels (Figure 6B) and fewer von Willebrand factor (vWF)-stained areas in the synovial tissues obtained from the fullerenol-injected joints compared with the tissues from the control joints (Figure 6C), thus increasing the evidence that the anti-angiogenesis effect is mediated by the down-regulated VEGF production resulting from fullerenol administration [19]. Collectively, these findings imply that the i.a. injection of fullerenol suppresses ROS formation and can ameliorate the rheumatism of joints by inhibiting pro-inflammatory cytokine production and the angiogenesis process.

A mouse model was used to examine the effect of systemic i.p. injection of fullerenol on the joints of mice with CIA. However, no differences were observed between the arthritis scores of the fullerenol- and PBS-injected mice through day 54 (Figure 7A), thus suggesting that the anti-arthritic effect is produced through a locally targeted mechanism rather than a systemic influence on the pathogenic environment. Next, we evaluated the anti-arthritis effect of fullerenol using the therapeutic protocol. The i.a. injected rat joints failed to demonstrate a therapeutic effect (Figure 7B), thus indicating that inhibiting additional mechanisms rather than ROS production alone might be required to suppress an actively inflamed rheumatoid joint. Finally, we examined the anti-arthritic effect of the i.a. injection of unmodified fullerene on the joints of rats with CIA. No effects were observed after using the prophylactic and therapeutic protocols (Figure 7C,D), confirming that aqueous solubility is required for such material to exert an in vivo pharmacological effect.

Although lowly hydroxylated fullerenol, C_60_(OH)_12–14_, is insoluble in water and exhibits no biological activity when introduced into a cell culture system, synthesized fullerenol with more hydroxyl groups has exhibited anti-viral and antioxidant activities for treating UV-induced injury of keratinocytes and experimental oncological models [8,20,21,22]. Notably, the two water-soluble hydroxylated fullerene derivatives—C_60_(OH)_32–34_ and C_60_(OH)_44_—have similar in vitro scavenging effects against free radicals [20]. Nevertheless, no studies have been published regarding the application of fullerenol for treating experimental models of autoimmune-related arthritis. In this study, the synthesized C_60_(OH)_36_ had in vitro anti-oxidative ability to reduce ROS production, and the direct i.a. administration resulted in reduced synovial expression of ROS and ameliorated the CIA in the joints. After systemic i.p. injection in another experimental model, non-modified fullerene exhibited a therapeutic effect against adjuvant-induced arthritis [23,24]. However, our experimental results failed to demonstrate the anti-arthritic effects of raw i.a. fullerene injection in CIA. Although different arthritis models and administration routes can cause discrepancies in the results of in vivo experiments, the aqueous solubility of injected materials may significantly influence the biological applications of fullerenes.

The therapeutic effect of fullerenol injection was not observed in the experimental CIA model in this study, and the effects of fullerenol appear to be limited to prophylactic intervention. This finding indicates that the inhibition of mechanisms other than ROS production may be required to suppress the established rheumatism in joints. Targeting synovial fibroblasts (SFs) is a novel approach that does not cause interference with the host’s defense, an inevitable side effect associated with the prevailing usage of biologics in RA patients [15,16]. Further studies can examine the effects of simultaneously targeting ROS and SFs in arthritis models. Interestingly, clinical observations have demonstrated a beneficial effect of reducing ROS production after co-administration of conventional RA medications and oral antioxidants, such as vitamin E and combined vitamins [25,26]. In particular, the i.a. injection, a method that avoids the adverse extra-articular reactions associated with systemic application, can provide improved bioavailability with lower drug costs compared with conventional methods [27]. According to the proof-of-concept results of this study, in the clinical scenario of RA patients with persistent monoarthritis refractory to standard oral therapy [14], the i.a. injection of fullerenol is a potential therapeutic modality. 

## 4. Conclusions

The i.a. injection of the water-soluble fullerenol C_60_(OH)_36_ synthesized in this study can ameliorate RA in joints by suppressing pro-inflammatory cytokine production and the angiogenesis process. Thus, the proposed method of targeting i.a. ROS production can be used as a pharmacological approach in RA.

## Figures and Tables

**Figure 1:** Illustrative graph of synthesized water-soluble fullerenol.

**Figure 2:** Timeline and procedure of collagen-induced arthritis (CIA) induction and treatment.

**Figure 3:** Functional characterization of the synthesized fullerenol. (**A**) Low-magnification TEM image shows the mean lateral size of a water-soluble fullerenol to be approximately 1.08 ± 0.03 nm (**B**) HR-TEM image of a water-soluble fullerenol illustrating the nanomaterials {$1\bar{1}00$} lattice planes and the mean size of 1.08 ± 0.03 nm with a *d*-spacing of 0.213 nm (inset: low-magnification TEM image of nanomaterials). (**C**) UV–Vis and (**D**) FTIR spectra of fullerenol. (**E**) Deconvoluted C(1s) X-ray photoelectron spectrometry (XPS) spectra and fitted peaks obtained using Gaussian function: nonoxygenated ring (C–C/C=C, 286.1 eV), C–OH bond (286.9 eV), and C–O^−^ bond (288.1 eV), respectively. The atomic ratio and bonding composition of fullerenol are shown as summarized in the table. The O(1s)/C(1s) atomic ratio is 37.1%.

**Figure 4:** Dose-dependent suppression of NO production obtained after treatment with various concentrations of fullerenol in the RAW 264.7 cell cultures.

**Figure 5:** Amelioration of CIA through the intra-articular (i.a.) injection of water-soluble C_60_(OH)_36_. (**A**) Articular indexes in the fullerenol- and PBS-injected CIA joints. (**B**) Nitrotyrosine-stained areas in synovial tissues obtained from fullerenol- and PBS-injected CIA joints with representative immunohistochemical staining. (**C**) Histological scores and representative hematoxylin and eosin (H&E)-stained synovial tissues obtained from the fullerenol- and PBS-injected CIA joints. (**D**) Radiological scores and representative radiographs of the fullerenol- and PBS-injected CIA joints. The values are the mean ± standard error of 16 joints per group in (**A**), 5 joints per group in (**B**), and 8 joints per group in (**C**,**D**). Bars represent 200 μm and 20 μm at 40× and 400×, respectively.

**Figure 6:** Amelioration of CIA by suppressing pro-inflammatory cytokine production and the angiogenesis process. (**A**) Interleukin (IL)-1β concentrations in joint extracts obtained from fullerenol- and PBS-injected CIA joints. (**B**) Vascular endothelial growth factor (VEGF) concentrations in joint extracts obtained from fullerenol- and PBS-injected CIA joints. (**C**) von Willebrand factor (vWF)-stained areas in synovial tissues obtained from fullerenol- and PBS-injected CIA joints, with representative immunohistochemical staining. The values are the mean ± standard error of 8 joints per group in (**A**,**B**), and 5 joints per group in (**C**). Bars represent 50 μm at 200×.

**Figure 7:** Arthritis scores after systemic administration, and articular indices of the therapeutic protocol and raw fullerene injection. (**A**) Mice with CIA that received the intraperitoneal (i.p.) injection of fullerenol or PBS. (**B**) Joints of rats with CIA after the i.a. injection of fullerenol or PBS using the therapeutic protocol. (**C**) Joints of rats with CIA after unmodified i.a. injection of fullerene or PBS using the prophylactic protocol. (**D**) Joints of rats with CIA after the i.a. injection of raw fullerene or PBS using the therapeutic protocol. The values of mean ± standard error are 10 mice per group in (**A**) and 16 joints per group in (**B**–**D**).

## Supplementary Materials

The following are available online at https://www.mdpi.com/2079-4991/9/6/909/s1, Figure S1: The size of water-soluble C_60_(OH)_36_ (fullerenol) was determined by the DLS and the average size was approximately 125.7 nm, which attributed to the hydrogen bond to form the aggregation of fullerenol.

## Abbreviations

ROS	reactive oxygen species
RA	rheumatoid arthritis
i.a.	intra-articular
CIA	collagen-induced arthritis
NO	nitric oxide
RIPA	radioimmunoprecipitation assay
IL	interleukin
VEGF	vascular endothelial growth factor
vWF	von Willebrand factor
i.p.	intraperitoneal
HR-TEM	high-resolution transmission electron microscope
UV–Vis	Ultraviolet–visible
FTIR	Fourier transform infrared
XPS	X-ray photoelectron spectrometry
LPS	Lipopolysaccharides
SPF	specific-pathogen-free
i.d.	intra-dermally
H&E	hematoxylin and eosin
ELISA	enzyme-linked immunosorbent assay
PBS	phosphate–buffered saline
TNF	tumor necrosis factor
SF	synovial fibroblast
